# MicroRNA-564 is downregulated in glioblastoma and inhibited proliferation and invasion of glioblastoma cells by targeting TGF-β1

This article has been retracted.

**DOI:** 10.18632/oncotarget.8987

**Published:** 2016-04-26

**Authors:** Chunming Jiang, Fang Shen, Jianmin Du, Zhaoyang Hu, Xiaoli Li, Jin Su, Xiaohua Wang, Xianmei Huang

**Affiliations:** ^1^ Department of Pediatrics, Affiliated Hangzhou Hospital of Nanjing Medical University, Hangzhou First People's Hospital, Hangzhou, Zhejiang 310003, P.R. China; ^2^ Department of Psychiatry, Tongde Hospital of Zhejiang Province, Hangzhou, Zhejiang 310012, P.R. China; ^3^ Translational Medicine Office of Hangzhou Cancer Institute, Affiliated Hangzhou Hospital of Nanjing Medical University, Hangzhou First People's Hospital, Hangzhou, Zhejiang 310003, P.R. China; ^4^ Department of Pediatrics, The First Affiliated Hospital of Nanjing Medical University, Nanjing, Jiangsu 210029, P.R. China; ^5^ Department of Pediatrics, Nanjing First Hospital, Nanjing Medical University, Nanjing, Jiangsu 210029, P.R. China

**Keywords:** glioblastoma, microRNA-564, TGF-β, proliferation

## Abstract

Increasing evidence has indicated that aberrant expression of miRNAs has been shown to be strongly implicated in the initiation and progression of glioblastoma. Here, we identified a novel tumor suppressive miRNA, miR-564, and investigated its role and therapeutic effect for glioblastoma. We showed that miR-564 was down-regulated in human glioblastoma tissues and cell lines. Introduction of miR-564 dramatically inhibited cell growth and invasion in glioblastoma cells. Subsequent experiments revealed that Transforming growth factor-β1 (TGF-β1) was a direct and functional target of miR-564 in glioblastoma cells. Furthermore, overexpression of miR-564 decreased p-SMAD and SMAD4 expression, which are the downstream signaling molecules of TGF-β. Meanwhile, ectopic of miR-564 reduced the messenger RNA (mRNA) and protein expression of epidermal growth factor receptor (EGFR) and MMP9. Furthermore, the upregulation of miR-564 suppressed TGF-β-mediated U87 proliferation and migration. The expression of EGFR and MMP9 was upregulated in glioblastoma tissues compared to their normal tissues. The EGFR and MMP9 expression levels were inverse correlated with the expression of miR-564. miR-564 suppressed the growth of U87-engrafted tumors. These findings reveal that miR-564/TGF-β1 signaling that may be required for glioblastoma development and may consequently serve as a new therapeutic target for the treatment of glioblastoma.

## INTRODUCTION

Glioblastoma is the most common and aggressive primary brain tumor and represent 12-15% of intracranial tumours and 60-75% of astrocytic tumours [1, 2]. Malignant gliomas account for approximately 70% of new cases of malignant primary brain tumors diagnosed in adults [3, 4]. This tumor is characterized by a high degree of invasiveness, rapid growth, and strong resistance to radiation and chemotherapy [5, 6]. Therefore, the prognosis for malignant gliomas has not significantly improved in the last four decades [7, 8]. To illuminate its complex characteristics, a gain deeper understanding of the molecular mechanisms underlying gliomagenesis is critical.

microRNAs (miRNAs) are 18–24 nucleotide, small non-coding, and evolutionarily conserved RNAs that posttranscriptionally regulate gene expression by binding to the 3-untranslated regions of target messenger RNAs [9–11]. Mature miRNAs can specifically bind to 3′UTRs of target cellular mRNA in turn triggering mRNA degradation or inhibition of translation [12, 13]. Accumulating studies have shown that miRNAs play important roles in a wide variety of biological processes, including development, cell proliferation, differentiation, apoptosis, metabolism, and signal transduction [14, 15]. It has been demonstrated that aberrant miRNAs expression correlates with various human cancers and indicates that miRNAs can function as oncogenes or tumor suppressor genes [16–19]. These findings suggest the miRNAs may play an important role in the pathogenesis of glioblastoma.

In our study, we have taken efforts to explore the potential roles of miR-564 in glioblastoma development. The expression of miR-564 in clinically human glioblastoma tissues and cell lines was evaluated. Furthermore, the roles of miR-564 in glioblastoma development and the underlying mechanisms were investigated. Our data indicate the roles of miR-564 in the control of cell growth and invasion in glioblastoma, and suggest the potential therapeutic application of miR-564 for glioblastoma patients.

## RESULT

### Reduced miR-564 expression in glioblastoma tissues and cell lines

qRT–PCR analysis has shown that the expression of miR-564 was decreased in all glioblastoma cell lines (U87, U251, LN229, A172, and U118) compared with NHAs, human Normal human astrocytes cell line (Figure 1A). We further quantified the expression level of miR-564 in 20 human glioblastoma tissues and 20 normal brain tissues (Figure 1B). The results also showed that the expression level of miR-564 was decreased in glioblastoma tissues compared with normal brain tissues.

**Figure 1:** Reduced miR-564 expression in glioblastoma tissues and cell lines **A.** Expression levels of miR-564 in normal human astrocytes (NHAs), 5 glioma cells (U87, U251, LN229, A172 and U118) was detected using qRT-PCR analysis. Transcript levels were normalized by U6 expression. **B.** qRT-PCR analysis of miR-564 expression in 20 pairs glioblastoma tissues and their corresponding nontumor glial brain tissues. The expression of miR-564 was normalized to U6 snRNA. ***p<0.001

### miR-564 Inhibits glioblastoma cell proliferation and invasion

We found that the expression of miR-564 was increased in transfected U87 cells using miR-564 mimics using qRT–PCR (Figure 2A). The CCK-8 proliferation assay showed that miR-564 inhibited the U87 cells proliferation (Figure 2B). The invasiveness of cells transfected with miR-564 mimics were decreased compared with the scramble group and untreat group cells (Figure 2C).

**Figure 2:** miR-564 Inhibits glioblastoma cell proliferation and invasion **A.** miR-564 mimics can enhance the expression of miR-564 in the U87 cells. **B.** The cells treated with miR-564 mimics or sramble or no transfection were measured by CCK8 assay at different time periods. **C.** Invasion analysis has shown that overexpression of miR-564 can repress the U87 cells invasion. The relative ratio of invasive cells per field is shown below, *p<0.05, ** p<0.01, and ***p<0.001.

### TGF-β1 is a direct target of miR-564

As illustrated in Figure 3A, the miRNA: mRNA alignment analysis showed that the 3′UTR of TGF-β1 contains one putative binding site for miR-564, located at 93–99 nt. Luciferase reporter gene assays showed that ectopic of miR-564 remarkably reduced luciferase activity in the TGF-β1 wild-type reporter gene but not the mutant TGF-β1 3′UTR, indicating that miR-564 directly targeted the TGF-β1 3′UTR (Figure 3B). Meanwhile, qRT–PCR analysis has shown that miR-564 overexpression repressed the mRNA expression of TGF-β; western blot analysis showed that ectopic expression of miR-564 markedly suppressed TGF-β protein expression in the U87 cell line (Figure 3C and 3D).

**Figure 3:** TGF-β1 is a direct target of miR-564 **A.** Predicted miR-564 target sequence in the 3′UTR of TGF-β1 (TGF-β1–3′-UTR-WT) and mutant containing 7 altered nucleotides in the 3′UTR of TGF-β1 (TGF-β1-3′-UTR-MUT). **B.** The analysis of the relative luciferase activities of TGF-β1-WT, TGF-β1-MUT in the U87 cells. **C.** qRT-PCR analysis of TGF-β1 mRNA expression in the U87 cells cells after treatment with miRNA mimics or scramble or no transfection. The expression of TGF-β1 was normalized to GAPDH. **D.** Western blot analysis of TGF-β1 expression in the U87 cells transfected with miR-564 mimics or scramble or no transfection. GAPDH was also detected as a loading control. ***p<0.001.

### MiR-564 overexpression repressed the p-SMAD, SMAD4, EGFR and MMP9 expression

Here, we conducted western blot to detect the downstream signaling molecules SMAD2, SMAD4, in the presence or absence of TGF-β, scramble, or miRNA-564, respectively. According to western blot results, SMAD4 and p-SMAD2 protein expression decreased with the treatment of miRNA-564 compared with scramble (Figure 4A). qRT–PCR analysis showed that TGF-β1 can enhance the mRNA and protein expression of MMP-9 and EGFR; meanwhile, following the miRNA-564 treatment, EGFR and MMP-9 proteins and mRNAs were significantly downregulated in the U87 cell line (Figure 4B, 4C and 4D).

**Figure 4:** MiR-564 overexpression repressed the p-SMAD, SMAD4, EGFR and MMP9 expression The U87 was treated in serum-free medium in the presence and absence of TGF-β1 (50 ng/ml), scramble, or miRNA-564 for 24 h. **A.** Expression of p-SMAD2, t-SMAD2 and SMAD4 was detected using western blotting. GAPDH was used as a loading control. **B.** The mRNA expression of MMP9 was detected using qRT-PCR. The expression of MMP9 was normalized to GAPDH. **C.** The mRNA Expression of EGFR was detected using qRT-PCR. The expression of EGFR was normalized to GAPDH. **D.** Expression of EGFR and MMP9 was detected using western blotting. GAPDH was used as a loading control.

### miR-564 is involved in TGF-β-induced tumor proliferation and invasion

The CCK-8 proliferation assay and invasion assay showed that TGF-β promoted the glioblastoma cell proliferation and invasion. When miR-564 mimic and TGF-β was added into U87 cells, miR-564 mimic inhibited the TGF-β -induced glioblastoma cell proliferation and invasion (Figure 5A and 5B).

**Figure 5:** miR-564 is involved in TGF-β-induced tumor proliferation and invasion The U87 was treated in serum-free medium in the presence and absence of TGF-β1 (50 ng/ml), scramble, or miRNA-564 for 24 h. **A.** Cell growth curves in U87 cells transfected with different combinations. **B.** Invasion analysis of U87 cells treated with different combinations. The relative ratio of invasive cells per field is shown right. *p<0.05, ** p<0.01, ***p<0.001.

### The expression of EGFR and MMP-9 was inversely expressed with miR-564

The expression of EGFR was upregulated in glioblastoma tissues compared to their normal tissues (Figure 6A). The expression of EGFR in glioblastoma tissues was significant higher than in normal brain tissues (Figure 6B). The EGFR expression levels were inverse correlated with the expression of miR-564 (Figure 6C, r^2^= −0.179; p<0.001). The expression of MMP9 was also upregulated in glioblastoma tissues compared to their normal tissues (Figure 6D). The expression of MMP9 in glioblastoma tissues was significant higher than in normal brain tissues (Figure 6E). The MMP9 expression levels were inverse correlated with the expression of miR-564 (Figure 6C, r^2^= −0.107; p<0.001).

**Figure 6:** The expression of EGFR and MMP9 was inversely expressed with miR-564 **A.** The expression of EGFR was measured by qRT-PCR. **B.** The expression of EGFR in glioblastoma tissues was significant higher than in normal brain tissues. **C.** The EGFR expression levels were inverse correlated with the expression of miR-564 (r^2^= −0.179; p<0.001). **D.** The expression of MMP9 was measured by qRT-PCR. **E.** The expression of MMP9 in glioblastoma tissues was significant higher than in normal brain tissues. **F.** The MMP9 expression levels were inverse correlated with the expression of miR-564 (r^2^= −0.107; p<0.001).

### miR-564 suppressed the growth of U87-engrafted tumors

We found that injection with miR-564 mimic suppressed the growth of U87-engrafted tumors compared to scrambled oligonucleotides-treated tumors (Figure 7A). The volumes and weights of tumor treated by miR-564 mimics were lower compared to scrambled mimics-injected tumors (Figure 7B and 7C). The mRNA and protein expression of TGF-β1 was lower in miR-564-treated tumors compared to the scramble-treated tumors (Figure 7D).

**Figure 7:** miR-564 suppressed the growth of U87-engrafted tumors **A.** Representative tumors were photographed treatment with miR-564 mimic or sramble. **B.** Graph representing tumor volumes at the indicated days during the experiment for the two groups: scrambled mimics, miR-564 mimics. **C.** Tumor weight averages between scrambled and miR-564 mimics-treated mice groups at the end of the experiment (day 25). **D.** The mRNA of TGF-β1 was measured by qRT-PCR. **E.** The protein of TGF-β1 was measured by western blot. *p<0.05, ** p<0.01, ***p<0.001.

## DISCUSSION

Glioblastoma is the most common type of malignant primary intracranial tumor and is characterized by the hallmarks of cellular heterogeneity, rapid proliferation, angiogenesis, extensive invasion, hypoxia and necrosis [20–22]. It is an urgent need to gain deeper understanding of molecular mechanisms implicated in glioblastoma progression and development [23]. Although miRNA signatures for glioblastoma have been established, eclucidation of the role of deregulated miRNAs in glioblastoma progression remains in the early stage of development. The data presented here showed a role of miR-564 in glioblastoma. In this study, we found that miR-564 were much lower in glioblastoma tissues compared with normal brain tissues. Furthermore, we showed that the restored expression of miR-564 in glioblastoma cell line U87 resulted in reduced cell proliferation and invasion. Moreover, we identified TGF-β1 as a direct target of miR-564. Furthermore, miR-564 overexpression can repress the expression of p-SMAD, SMAD4, EGFR and MMP9, which are the downstream signaling molecules of TGF-β. miR-564 is also involved in TGF-β-induced tumor proliferation and invasion. The expression of EGFR and MMP9 was upregulated in glioblastoma tissues compared to their normal tissues. The EGFR and MMP9 expression levels were inverse correlated with the expression of miR-564. miR-564 suppressed the growth of U87-engrafted tumors. Our findings, together with those other groups, suggest that miR-564 has a fundamental role in glioblastoma tumorigenesis and cell invasion.

Previous study has reported that miR-564 were down-regulated in chronic myeloid leukemia cells [24]. However, the expression and function of miR-564 in glioblastoma remains to be determined. Our results have been shown that miR-564 was down-regulated in glioblastoma tissues compared with normal brain tissues. Moreover, restoration of miR-564 can reduce glioblastoma cell proliferation and invasion. Although effective delivery of miRNA mimic into the brain, crossing the blood-brain barrier, remains challenging, the striking inhibitory effect of miR-564 on cell growth and invasion strongly suggests that further efforts toward development of miR-564-based therapeutics are fully warranted.

Recently, TGF-β has been shown to promote tumor progression and invasion by TGF-β signaling pathway in glioblastoma, especially in high-grade gliomas [25, 26]. TGF-β activates a heterodimeric complex including TβR-I and TβR-II and initiates a signaling cascade through phosphorylation of the specific receptor regulated SMAD2/3 [21]. Similarly, the non-SMAD dependent signaling regulated by TGF-β is also believed to be crucial in tumor progression [27, 28]. Therefore, TGF-β signaling pathway has been considered a therapeutic target due to its involvement in cell proliferation and epithelial mesenchymal transition in glioblastoma [25, 29, 30]. However, the underlying mechanisms are unclear. Our data showed that the ability of miR-564 to target TGF-β1 may provide one such mechanism of post-transcriptional control of TGF-β1. This conclusion is supported by the following reasons: complementary sequence of miR-564 is identified in the 3′UTR of TGF-β1 mRNA; reintroduction of miR-564 led to a significant reduction in reintroduction at both mRNA and protein level; overexpression of miR-564 suppressed reintroduction 3′UTR luciferase report activity and this effect was abolished by mutation of the miR-564 seed binding site. These results indicate that miR-564 may function as a tumor suppressor partly mediated by repressing TGF-β1 expression in glioblastoma development.

We further studied the functional roles of miRNA-564 in TGF-β signaling pathways. In the present study, we have shown that TGF-β can induce the p-SMAD and SMAD4 expression. Moreover, the forced miRNA-564 inhibited the p-SMAD and SMAD4 expression. Previous studies reported that TGF-β can induce the EGFR and MMP9 expression [21]. In line with this result, our result also has shown that TGF-β can induce the EGFR and MMP9 expression. Our data demonstrated that miRNA-564 overexpression affected TGF-β-induced EGFR and MMP9 expression in the U87 cells. Since EGFR and MMP9 regulate glioblastoma cell proliferation, survival, migration, and invasion and plays a key role in tumor progression. Furthermore, overexpression of miR-564 is involved in TGF-β-induced tumor proliferation and invasion.

In conclusion, the identification of miR-564 as a tumor suppressive miRNA in human glioblastoma that acts by repressing TGF-β1 provides additional evidence of a pivotal role for miRNAs in glioblastoma progression. Given that miR-564 is downregulated in glioblastoma, the introduction of this mature miRNA into the tumor tissue could serve as a therapeutic strategy by reducing the expression of target genes. MiRNA-based therapeutic patterns are still in their infancy; however, our findings are encouraging and suggest that this miRNA could be targeted for the development of a treatment for patients with glioblastoma in the future.

## MATERIALS AND METHODS

### Ethics statement

All patients or patients'parents on behalf of the children agreed to participate in the study and gave written informed consent. This study and consent was approved by the ethical board of the institute of Tangde Hospital and Hangzhou First People's Hospital complied with Declaration of Helsinki.

### Human tissue

Glioblastoma samples were obtained from the Tongde Hospital, Hangzhou First People's Hospital and The First Affiliated Hospital of Nanjing Medical University from 2013 to 2014. The histological features of all specimens were confirmed by pathologists according to the WHO criteria. None of the patients had received radiotherapy or chemotherapy before tumor resection. Normal brain tissues were taken from peripheral nontumor glial brain tissue from the same patient.

### Cell lines and culture

Human GBM cell lines U87, U251, LN229, A172, and U118 were purchased from the American Type Culture Collection (ATCC, Manassas, Va.) and grown in Dulbecco's modified Eagle's medium (DMEM) supplemented with 10% fetal bovine serum (FBS). Normal human astrocytes (NHAs) were purchased from Lonza and cultured in the provided astrocyte growth media supplemented with rhEGF, insulin, ascorbic acid, GA-1000, L-glutamine and, 5% FBS.

### RNA extraction and real-time quantitative PCR

Total RNA was extracted from tissues or the cells using Trizol (Invitrogen) according to the manufacturer's protocol. The expression of miR-564 was measure by quantitative RT-PCR (qRT-PCR) with the TaqMan microRNA assays reverse transcription kit according to the manufacturer's instructions (Applied Biosystems, Foster City, CA). The expression of U6 was used as internal control. Real-time PCR was performed on a Real-Time PCR System (Applied Biosystems, Foster City, CA) in duplicates. The difference of CT values between internal control and miR-564 was presented as −ΔCT. ΔΔCT is the difference of ΔCT values between paired specimens. 2^ΔΔCT^ represents the exponential value of ΔCT, which means fold change in expression. The mRNA expression of GAPDH was used as internal control.

### Oligonucleotide transfection

The miR-564 mimics and scramble were synthesized by GenePharma (Shanghai, China) and transfected into the cells to a final oligonucleotide concentration of 20 nmol/L. All cell transfections were introduced by Lipofectamine 2000 (Invitrogen) according to the manufacturer's instructions.

### Western blotting

Total protein was extracted from frozen tissues or the cells using a Total Protein Extraction Kit (KeyGen, Nanjing, China) according to the manufacturer's instructions. Protein concentration was confirmed by the Bradford assay. Protein was separated by 10% SDS-PAGE and then transferred to PVDF membrane using standard procedures. The membrane was incubated with the primary antibody for TGF-β1 (Sigma, St. Louis, MO) or GAPDH (Cell Signaling Technology, Beverly, MA, USA), and then washed, incubated with HRP-conjugated secondary antibody. Intensity of the bands was visualized by an enhanced chemiluminescence (ECL, Amersham Pharmacia Biotech) system and exposed.

### Cell proliferation and migration assays

Cell proliferative activity was determined by the Cell Counting Kit-8 (CCK-8; Dojindo, Kumamoto, Japan) assay, according to standard methods. Absorbance was measured at 450 nm and detected using μQuant Universal Microplate Spectrophotometer (BioTek Instruments, Inc.). For analysis of cell invasion, the transwell chambers were coated with Matrigel (BD Biosciences, San Jose, CA, USA) and incubated at 37 °C for 2 h, allowing it to solidify. After 24 h of transfection, 4×10^5^ cells suspended in serum-free DMEM were added to the upper chamber, and medium containing 10 % FBS was added to the lower chamber. After 24 h, invasive cells located on the lower surface of the chamber were stained.

### Dual luciferase reporter assay

The wild-type (WT) and mutated putative miR-564 target on TGF-β1 3′UTR were cloned into the pGL3 Dual-Luciferase miRNA Target Expression Vector (Invitrogen Corporation). Luciferase activity was measured with the dual luciferase reporter assay system (Promega) according manufacturer's instructions.

### Xenograft tumor assay

Female nude mice were injected subcutaneously with U87. MiR-564 mimic or scramble oligonucleotide was injected into the tumors when directly injected into the tumors. The tumor including length, width and weight was measured every three days. Mice were killed on the 25th days after injection.

### Statistic analysis

Data were presented as the mean ± standard deviation (SD) from three separate experiments. The differences between groups were analyzed using Student's t-test when only two groups were compared or a one-way analysis of variance (ANOVA) when more than two groups were compared. The differences between groups of metastasis in vivo were analyzed using the χ2 test. All of the statistical analyses were performed with SPSS 16.0 (SPSS Inc., USA). The difference was considered to be statistically significant at P<0.05.

## SUPPLEMENTARY MATERIALS TABLE



## References

[1] Hiddingh L, Tannous BA, Teng J, Tops B, Jeuken J, Hulleman E, Boots-Sprenger SH, Vandertop WP, Noske DP, Kaspers GJ, Wesseling P, Wurdinger T (2014). EFEMP1 induces gamma-secretase/Notch-mediated temozolomide resistance in glioblastoma. Oncotarget.

[2] Goldshmit Y, Trangle SS, Kloog Y, Pinkas-Kramarski R (2014). Interfering with the interaction between ErbB1, nucleolin and Ras as a potential treatment for glioblastoma. Oncotarget.

[3] Guo J, Shinriki S, Su Y, Nakamura T, Hayashi M, Tsuda Y, Murakami Y, Tasaki M, Hide T, Takezaki T, Kuratsu J, Yamashita S, Ueda M, Li JD, Ando Y, Jono H (2014). Hypoxia suppresses cylindromatosis (CYLD) expression to promote inflammation in glioblastoma: possible link to acquired resistance to anti-VEGF therapy. Oncotarget.

[4] Srinivasan S, Patric IR, Somasundaram K (2011). A ten-microRNA expression signature predicts survival in glioblastoma. PloS one.

[5] Chan JA, Krichevsky AM, Kosik KS (2005). MicroRNA-21 is an antiapoptotic factor in human glioblastoma cells. Cancer research.

[6] Dong H, Luo L, Hong S, Siu H, Xiao Y, Jin L, Chen R, Xiong M (2010). Integrated analysis of mutations, miRNA and mRNA expression in glioblastoma. BMC systems biology.

[7] Novakova J, Slaby O, Vyzula R, Michalek J (2009). MicroRNA involvement in glioblastoma pathogenesis. Biochemical and biophysical research communications.

[8] D'Urso PI, D'Urso OF, Storelli C, Mallardo M, Gianfreda CD, Montinaro A, Cimmino A, Pietro C, Marsigliante S (2012). miR-155 is up-regulated in primary and secondary glioblastoma and promotes tumour growth by inhibiting GABA receptors. International journal of oncology.

[9] Li M, Yu M, Liu C, Zhu H, He X, Peng S, Hua J (2013). miR-34c works downstream of p53 leading to dairy goat male germline stem-cell (mGSCs) apoptosis. Cell proliferation.

[10] Huang J, Zhang SY, Gao YM, Liu YF, Liu YB, Zhao ZG, Yang K (2014). MicroRNAs as oncogenes or tumour suppressors in oesophageal cancer: potential biomarkers and therapeutic targets. Cell proliferation.

[11] Li J, You T, Jing J (2014). MiR-125b inhibits cell biological progression of Ewing's sarcoma by suppressing the PI3K/Akt signalling pathway. Cell proliferation.

[12] Ohdaira H, Sekiguchi M, Miyata K, Yoshida K (2012). MicroRNA-494 suppresses cell proliferation and induces senescence in A549 lung cancer cells. Cell proliferation.

[13] Li Z, Lei H, Luo M, Wang Y, Dong L, Ma Y, Liu C, Song W, Wang F, Zhang J, Shen J, Yu J (2015). DNA methylation downregulated mir-10b acts as a tumor suppressor in gastric cancer. Gastric cancer.

[14] Yu X, Li Z (2014). MicroRNAs regulate vascular smooth muscle cell functions in atherosclerosis (review). International journal of molecular medicine.

[15] Yu X, Li Z, Shen J, Wu WK, Liang J, Weng X, Qiu G (2013). MicroRNA-10b Promotes Nucleus Pulposus Cell Proliferation through RhoC-Akt Pathway by Targeting HOXD10 in Intervetebral Disc Degeneration. PloS one.

[16] Bier A, Giladi N, Kronfeld N, Lee HK, Cazacu S, Finniss S, Xiang C, Poisson L, de Carvalho AC, Slavin S, Jacoby E, Yalon M, Toren A, Mikkelsen T, Brodie C (2013). MicroRNA-137 is downregulated in glioblastoma and inhibits the stemness of glioma stem cells by targeting RTVP-1. Oncotarget.

[17] Perilli L, Vicentini C, Agostini M, Pizzini S, Pizzi M, D'Angelo E, Bortoluzzi S, Mandruzzato S, Mammano E, Rugge M, Nitti D, Scarpa A, Fassan M, Zanovello P (2014). Circulating miR-182 is a biomarker of colorectal adenocarcinoma progression. Oncotarget.

[18] Zhang C, Liu J, Wang X, Wu R, Lin M, Laddha SV, Yang Q, Chan CS, Feng Z (2014). MicroRNA-339-5p inhibits colorectal tumorigenesis through regulation of the MDM2/p53 signaling. Oncotarget.

[19] Bier A, Giladi N, Kronfeld N, Lee HK, Cazacu S, Finniss S, Xiang C, Poisson L, deCarvalho AC, Slavin S, Jacoby E, Yalon M, Toren A, Mikkelsen T, Brodie C (2013). MicroRNA-137 is downregulated in glioblastoma and inhibits the stemness of glioma stem cells by targeting RTVP-1. Oncotarget.

[20] Lukiw WJ, Cui JG, Li YY, Culicchia F (2009). Up-regulation of micro-RNA-221 (miRNA-221; chr Xp11. 3) and caspase-3 accompanies down-regulation of the survivin-1 homolog BIRC1 (NAIP) in glioblastoma multiforme (GBM). Journal of neuro-oncology.

[21] Lv S, Sun B, Dai C, Shi R, Zhou X, Lv W, Zhong X, Wang R, Ma W (2015). The Downregulation of MicroRNA-146a Modulates TGF-beta Signaling Pathways Activity in Glioblastoma. Mol Neurobiol.

[22] Zhang R, Luo H, Wang S, Chen W, Chen Z, Wang HW, Chen Y, Yang J, Zhang X, Wu W, Zhang SY, Shen S, Dong Q, Zhang Y, Jiang T, Lu D (2014). MicroRNA-377 inhibited proliferation and invasion of human glioblastoma cells by directly targeting specificity protein 1. Neuro-oncology.

[23] Tanase C (2013). miRNA interactions as a novel molecular panel for clinical outcome of glioblastoma. Biomarkers in medicine.

[24] Rokah OH, Granot G, Ovcharenko A, Modai S, Pasmanik-Chor M, Toren A, Shomron N, Shpilberg O (2012). Downregulation of miR-31, miR-155, and miR-564 in chronic myeloid leukemia cells. PloS one.

[25] Seystahl K, Tritschler I, Szabo E, Tabatabai G, Weller M (2015). Differential regulation of TGF-beta-induced, ALK-5-mediated VEGF release by SMAD2/3 versus SMAD1/5/8 signaling in glioblastoma. Neuro Oncol.

[26] Lv S, Zhang J, Han M, Wang W, Zhang Y, Zhuang D, Shi R, Bian R, Yao C (2015). Nucleolin Promotes TGF-beta Signaling Initiation via TGF-beta Receptor I in Glioblastoma. J Mol Neurosci.

[27] Lin B, Madan A, Yoon JG, Fang X, Yan X, Kim TK, Hwang D, Hood L, Foltz G (2010). Massively parallel signature sequencing and bioinformatics analysis identifies up-regulation of TGFBI and SOX4 in human glioblastoma. PloS one.

[28] Zhang Z, Wu L, Wang J, Li G, Feng D, Zhang B, Li L, Yang J, Ma L, Qin H (2014). Opposing effects of PI3K/Akt and Smad-dependent signaling pathways in NAG-1-induced glioblastoma cell apoptosis. PloS one.

[29] Joseph JV, Conroy S, Tomar T, Eggens-Meijer E, Bhat K, Copray S, Walenkamp AM, Boddeke E, Balasubramanyian V, Wagemakers M, den Dunnen WF, Kruyt FA (2014). TGF-beta is an inducer of ZEB1-dependent mesenchymal transdifferentiation in glioblastoma that is associated with tumor invasion. Cell death & disease.

[30] Jiang H, Jin C, Liu J, Hua D, Zhou F, Lou X, Zhao N, Lan Q, Huang Q, Yoon JG, Zheng S, Lin B (2014). Next generation sequencing analysis of miRNAs: MiR-127-3p inhibits glioblastoma proliferation and activates TGF-beta signaling by targeting SKI. Omics.

